The article "Retinoic acid combined with spermatogonial stem cell conditions facilitate the generation of mouse germ-like cells" was published in 2017. Journal: Biosci Rep.

# Retinoic acid combined with spermatogonial stem cell conditions facilitate the generation of mouse germ-like cells

**DOI:** 10.1042/BSR20170637

**Published:** 2017-04-20

**Authors:** Guoyi Dong, Zhouchun Shang, Longqi Liu, Chuanyu Liu, Yuping Ge, Quanlei Wang, Liang Wu, Fang Chen, Baolin Li, Xin Liu, Xun Xu, Huanming Yang, Yutao Du, Hui Jiang

**Affiliations:** 1 BGI-Shenzhen, Shenzhen, China; 2 Department of Regenerative Medicine, Tongji University School of Medicine, Shanghai 200092, China; 3 Shenzhen Engineering Laboratory for Innovative Molecular Diagnostics, BGI-Shenzhen, Shenzhen, China; 4 Section of Molecular Disease Biology, Department of Veterinary Disease Biology, Faculty of Health and Medical Sciences, University of Copenhagen, Copenhagen, Denmark; 5 James D. Watson Institute of Genome Sciences, Hangzhou, China

**Keywords:** Differentiation, Germ-like cells, Retinoic acid, Spermatogonial stem cell conditions

## Abstract

Spermatogenic lineage has been directly generated in spermatogonial stem cell (SSC) conditions from human pluripotent stem cells (PSCs). However, it remains unknown whether mouse embryonic stem cells (ESCs) can directly differentiate into advanced male germ cell lineage in the same conditions. Here, we showed rather low efficiency of germ-like cell generation from mouse ESCs in SSC conditions. Interestingly, addition of retinoic acid (RA) into SSC conditions enabled efficient differentiation of mouse ESCs into germ-like cells, as shown by the activation of spermatogenesis-associated genes such as *Mvh*, *Dazl*, *Prdm14*, *Stella*, *Scp1*, *Scp3*, *Stra8* and *Rec8*. In contrast, for cells cultured in control medium, the activation of the above genes barely occurred. In addition, RA with SSC conditions yielded colonies of Acrosin-expressing cells and the positive ratio reached a peak at day 6. Our work thus establishes a simple and cost-efficient approach for male germ like cell differentiation from mouse PSCs and may propose a useful strategy for studying spermatogenesis *in vitro.*

## Introduction

Infertility, caused by the absence or disruption of germ cells, is becoming a significant human health concern because it affects 10–15% couples [1]. A potentially useful treatment to restore non-genetically caused male infertility is the stem cell transplantation using primordial germ cells (PGCs) or advanced germ cells [2–4]. PGCs, the precursors of gametes, originate from post-implantation epiblast cells and are established *in vivo* through extracellular cytokines in extraembryonic tissues [5]. Researchers have now successfully produced PGCs from pluripotent stem cells (PSCs) *in vitro* through activating a number of key signals, such as bone morphogenetic proteins (BMP2, BMP4 and BMP8B) [6] or genetic means by inducing ectopic expression of PGCs-specific transcription factors (BLIMP1, PRDM14 and AP2γ). Moreover, engineering PGCs using mouse PSCs are able to differentiate into advanced germ cells including gametes through transplantation in mice *in vivo* [7,8] or even differentiate into functional haploid spermatid-like cells *in vitro* [9]. These findings suggest that conversion of PSCs into gametes is now possible.

The article "Retinoic acid combined with spermatogonial stem cell conditions facilitate the generation of mouse germ-like cells" was published in 2017. Journal: Biosci Rep.

However, one major challenge in this field is how to directly and efficiently differentiate PSCs into post-meiotic, haploid germ cells *in vitro*. Kee et al. [10] firstly showed the direct differentiation of human embryonic stem cells (ESCs) into haploid germ cells through ectopic expression of *DAZL, DAZ* and *BOULE* genes. The same method was applied later to human induced PSCs (iPSCs) [11,12]. However, the introduction of exogenous factors brings genetic modifications that could raise risks for further clinical applications. In this regard, Easley et al. [13] firstly showed direct and efficient generation of haploid spermatogenic cells from human ESCs and iPSCs in spermatogonial stem cell (SSC) conditions, which provides a promising method to directly obtain spermatid-like cells without genetic manipulation.

Previous reports showed that retinoic acid (RA), a derivative of vitamin A, plays important roles in embryogenesis and cellular differentiation [14,15]. Interestingly, RA can also promote spermatogenesis through activation of key genes that initiates meiosis [16–19]. In addition, vitamin A deficient (VAD) male mice showed spermatogonia deficiency [20]. These evidence indicate that RA is an important player during gametogenesis.

Since SSC conditions can directly and efficiently generate haploid spermatogenic cells from human ESCs [13], whether it also works for mouse ESCs differentiation or whether adding RA into SSC conditions could enhance the induction efficiency of mouse spermatogenic linage differentiation would be an interesting questions, because mouse ESCs represent naïve pluripotency state which is distinct from primed state of human ESCs or iPSCs [21], and is a widely used model to study germ cell specification [7,22–25]. Considering recent advances in the establishment of human naïve PSCs [26–29], generation of germ cells directly from naïve PSCs would help the clinical application of human naïve PSCs.

In the present study, we demonstrated that mouse spermatogenic cell specification in SSC conditions showed extremely low efficiency, which was distinct from that in humans. We then found that RA combined with SSC conditions significantly enhanced mouse ESCs differentiation efficiency through increasing the expression of spermatogenic genes. We further identified Acrosin-positive cells in SSC conditions with RA. Thus, our findings partially contribute to the goal of understanding germ cell development *in vitro*.

The article "Retinoic acid combined with spermatogonial stem cell conditions facilitate the generation of mouse germ-like cells" was published in 2017. Journal: Biosci Rep.

## Materials and methods

### Ethical statement

All animal experiments were performed under the Guide for the Care and Use of Laboratory Animals in BGI.

### Cell culture

Briefly, human iPSCs (hiPSCs-99-2) were generated from dermal fibroblasts (Fib-99) of a 26-year-old male by overexpression of the Yamanaka factors *OCT3/4*, *SOX2*, *KLF4* and *c-MYC*, as described previously [30]. hiPSCs-99-2 and ESCs (H1) were maintained on feeder in standard medium contained DMEM/F12 (Gibco, 11320-033), 20% KSR (Gibco, 10828-028), 2 μM L-glutamine (Sigma, G8540), 0.1 μM NEAA (Gibco, 11140-050), 0.1 μM 2-Mercaptoethanol (Gibco, 21985-023) and 10 ng/ml human bFGF (Invitrogen, PHG0021). Mouse ESCs were isolated and cultured in mouse ESC medium containing DMEM/F12 (Gibco, 11320-033), 20% KSR (Gibco, 10828-028), 1 μM sodium pyruvate (Sigma, 10828), 2 μM L-glutamine (Sigma, G8540), 0.1 μM NEAA (Gibco, 11140-050), 0.1 μM 2-Mercaptoethanol (Gibco, 21985-023) and 10 ng/ml LIF (Millipore, LIF1010). The medium was replaced daily. Male ESCs lines were identified by PCR using *Sry* gene.

### Human and mouse spermatogenic lineage differentiation

SSC differentiation assays were performed as described previously [13]. Briefly, human ESCs (H1)/iPSCs (hiPSCs-99-2) and mouse ESCs were digested and transferred to matrigel coated 24-well plates (BD, 356231) and maintained for 3 days. Then the medium was changed to SSC conditions with or without RA (2 μM, R2625), the medium was replaced daily (Figure 1A). The SSC conditions contained (all from Sigma, unless otherwise noted) minimum essential medium (MEM) α (Invitrogen, 12571-063), 0.2% BSA (Invitrogen, 11020021), 5 mg/ml insulin (Wako, 093-06471), 10 mg/ml transferrin (T8158), 60 mM putrescine (P5780), 2 mM L-glutamine (Invitrogen, 25030-149), 50 mM b-mercaptoethanol (M3148), 1 ng/ml human bFGF (Invitrogen, PHG0021), 20 ng/ml glial cell line-derived neurotrophic factor (GDNF) (R&D Systems, 212-GD-010), 30 nM sodium selenite (S9133), 2.36 mM palmitic acid (P5585), 0.21 mM palmitoleic acid (P9417), 0.88 mM stearic acid (S4751), 1.02 mM oleic acid (01383), 2.71 mM linoleic acid (L1012), 0.43 mM linolenic acid (L2376), 10 mM HEPES (H3784) and 0.5× penicillin/streptomycin (V900929).

**Figure 1:** Human and mouse PSCs show distinct differentiation potential towards spermatogenic lineage in SSC conditions (**A**) A schematic illustration of the differentiation procedure. (**B**) Morphology and alkaline phosphatase (AP) staining of hESCs-H1, hiPSCs-99-2 and mouse ESCs (mESCs) respectively. Scale bar, 100 μm. (**C**,**D**) Immunofluorescence staining with MVH (C) and DAZL (D) at day 6 (mouse) and day 10 (human) of PSCs differentiation in SSC conditions. Scale bar, 100 μm.

The article "Retinoic acid combined with spermatogonial stem cell conditions facilitate the generation of mouse germ-like cells" was published in 2017. Journal: Biosci Rep.

### Reverse transcription and quantitative real-time PCR

Cells were collected at day 0, 3, 5 and 6 and lysed by TRIzol. Total RNA was extracted using isolation reagent (Invitrogen, 10296-028) according to the manufacturer’s instructions. Three micrograms of total RNA was used for reverse transcription through the Prime Script First Strand cDNA Synthesis Kit (Takara, D6110A). Quantitative real-time PCR (QPCR) was performed using SYBR (Takara, RR420A). Primers for QPCR analyses are shown in Table 1.

**Table 1:** Primers used for QPCR analysis

Gene	Forward	Reverse
*Oct4*	GCAGATCACTCACATCGCCA	GTAGCCTCATACTCTTCTCGTTGG
*Nanog*	TTACAAGGGTCTGCTACTGA	TTTGGGACTGGTAGAAGAAT
*Sox2*	CTCCATGACCAGCTCGCAGAC	GGCCTCGGACTTGACCACAG
*Dazl*	AATGTTCAGTTCATGATGCTGCTC	TGTATGCTTCGGTCCACAGACT
*Mvh*	TATGATGCGGGATGGAAT	CACCCTTGTACTATCTGTCG
*Prdm14*	ACAGCCAAGCAATTTGCACTAC	TTACCTGGCATTTTCATTGCTC
*Stella*	AGGCTCGAAGGAAATGAGTTT	TCCTAATTCTTCCCGATTTTCG
*Plzf*	CGCCACCTTCGCTCACAT	TGAACCCTGTAGTGCGTCTC
*Scp1*	CGCTACAACCACATGCTTCG	GGAACGCTGCTTAGATCTCCTC
*Scp3*	AGCAGAGAGCTTGGTCGGG	TCCGGTGAGCTGTCGCTGTC
*Stra8*	GTTTCCTGCGTGTTCCACAAG	GTTTCCTGCGTGTTCCACAAG
*Rec8*	AAGAATGCTCAGACAAAGGCCA	CGATCTCGCTCAGAGCTTCAGT
*acrosin*	GAAACAAGCCAGTGAAAGA	CAGCAGGGTCCAATGAAG
*Sry*	GTGGTCCCGTGGTGAGA	AACAGGCTGCCAATAAA
*β-Actin*	AGAGGGAAATCGTGCGTGAC	CAATAGTGATGACCTGGCCG

### AP and immunofluorescence staining

AP staining was performed using the Leukocyte Alkaline Phosphatase kit (Sigma, AM0100). For immunofluorescence staining, differentiated cells at each time points were fixed in methanol for 5 min, then cells were washed with PBS and permeabilized with 0.25% Triton X-100 in PBS for 10 min. Then cells were blocked using 1% BSA (Invitrogen, 11020021) for 30 min. The primary antibodies against SOX2 (Abcam, ab75485), MVH (Abcam, ab13840), DAZL (Abcam, ab34139) and Acrosin (Santa Cruz, sc-46284) were diluted at 1:100 and incubated for overnight at 4°C. On the second day, cells were then stained with FITC anti-rabbit secondary antibody (Santa Cruz, sc-2012) or Cy3 IgG secondary antibody (Abcam, ab6939) for 1 h at room temperature (RT), cells were washed with PBS and stained with DAPI for 5 min at RT. Finally, cells were mounted with mineral oil and examined under fluorescence microscopy.

### FACS analysis of Acrosin-positive cells

Differentiated cells at day 6 were dissociated with 0.25% trypsin, neutralized with DMEM containing 10% FBS, then washed twice with PBS and fixed with 4% paraformaldehyde for 30 min at RT and then rinsed twice with PBS. The fixed cells were permeabilized with 0.25% Triton X-100 in PBS for 10 min and washed with PBS again. The cells were blocked with 1% BSA in PBS for 30 min at RT and then incubated with PE–conjugated rabbit Acrosin antibody for 1 h at RT. The cells were resuspended in PBS, and analysed by using FACS Calibur (BD Biosciences) after two washes. Normal mouse ESCs were used as control.

The article "Retinoic acid combined with spermatogonial stem cell conditions facilitate the generation of mouse germ-like cells" was published in 2017. Journal: Biosci Rep.

### Statistical analysis

Results were given as mean ± S.E.M. and statistically significant differences (*P*<0.05) were determined by ANOVA analysis using GraphPad Prism 5 and FlowJo 7.6.1 software.

## Results

### Human and mouse ESCs show distinct differentiation potential towards germ-like cells in SSC conditions

Human ESCs (H1) and hiPSCs-99-2 were subjected to differentiate into spermatogenic cell for validating the induction system. Colonies from both cell lines showed normal morphology and were AP staining positive (Figure 1B). We then used the strategy of Easley et al. [13] to differentiate both cell lines into spermatogenic lineage in SSC conditions. Consistent with previous results, we observed the appearance of advanced germ-like cells during the differentiation process, as shown by the immunofluorescence staining of MVH and DAZL, two markers for premeiotic spermatogonia cells (Figure 1C,D), suggesting that this system is reproducible and could be used for further study.

Next, we performed mouse ESCs differentiation towards spermatogenic lineage in SSC conditions. We isolated mouse ESCs from a mouse strain (Figure 1B). We then cultured mouse ESCs in SSC conditions and performed spermatogonia differentiation using the same strategy as in human PSCs. Surprisingly, we observed almost no MVH- or DAZL-positive colonies during this process (Figure 1C,D).

### RA promotes the generation of germ-like cells in SSC conditions

We performed mouse ESCs differentiation assay in SSC conditions with or without RA. Different time points of samples were collected and expression for genes related to spermatogenic differentiation was measured by QPCR. Surprisingly, an increasing gene expression of *Mvh* and *Dazl* at first day 3 and then a maximum at day 6 in SSC conditions with RA was observed. The increasing level of *Mvh* and *Dazl* were significantly different at day 3 and day 6 respectively compared with that in SSC conditions (*, *P*<0.05; **, *P*<0.01, Figure 2A).

**Figure 2:** RA promotes the generation of germ-like cells in SSC conditions (**A**) Expression of *Mvh* and *Dazl* at day 3 and day 6 during mESCs differentiation in SSC conditions with or without RA. Values with * show significant differences among different treatments at the indicated time points (*, *P*<0.05; **, *P*<0.01; ***, *P*<0.001). (**B**,**C**) Immunofluorescence staining with SOX2, MVH and DAZL at day 3 and day 6 during mESCs differentiation in SSC conditions with or without RA. Scale bar, 100 μm.

The article "Retinoic acid combined with spermatogonial stem cell conditions facilitate the generation of mouse germ-like cells" was published in 2017. Journal: Biosci Rep.

To further specify the spermatogenic lineage differentiation, we analysed the protein expression of mouse MVH, a specific protein for differentiating germ cells and DAZL, a key intrinsic factor stimulating translation of MVH and response to extrinsic RA [16,31]. As expected, our results showed that MVH and DAZL were detected at day 3 and highly expressed in SSC conditions with RA at day 6 (Figure 2B,C). Therefore, our data suggest that RA facilitates the differentiation of mouse ESCs into spermatogenic lineage in SSC conditions.

To test whether cells undergo the progress of PGCs stage in SSC condition with RA, we analysed two PGCs markers, *Prdm14* and *Stella*. As expected, the expressions of these two genes were notably increased from day 5 to day 6 (Figure 3A,B). In addition, the expression of *Sox2* in SSC conditions with RA was slightly decreased at day 3, and then increased from day 3 to 6 (Figure 3C). Together, our results indicated that cells undergo a differentiation progress of PGCs stage.

**Figure 3:** Elevated spermatogenic gene expression during mESCs differentiation (**A**–**J**) QPCR results of *Prdm14* (A), *Stella* (B), *Sox2* (C), *Plzf* (D), *Scp1* (E), *Scp3* (F), *Stra8* (G), *Rec8* (H), *Oct4* (I), *Nanog* (J) expression at day 0, 3, 5 and 6 during mouse ESCs differentiation in SSC conditions with or without RA. The expression levels of mRNA were normalized to *β-actin*, and expressed as a ratio of mRNA levels of genes of interest to that of *β-actin*. The values of the three replicates were given as the mean ± S.D. Values with * show significant differences among different treatments at the indicated time points (*, *P*<0.05; **, *P*<0.01; ***, *P*<0.001).

To investigate whether meiosis happens in the case of our differentiation process, we then focused on the gene expression dynamics for several genes, *Plzf*, which plays critical roles in the SSC self-renewal [32]; *Stra8* and *Rec8*, which regulate the meiotic initiation [18,33]; *Scp1* and *Scp3*, which are required for synapsis phase of meiosis [34,35]. We measured their expression level at different time points during differentiation by QPCR (Figure 3D–H). As expected, we observed the expression of *Plzf*, *Rec8* and *Scp3* genes remarkably increased at later time points. In contrast, we observed elevated expression of *Stra8* and *Scp1* at an early stage and decreased at later time points. Furthermore, our QPCR results (Figure 3G) showed that the expression of *Stra8* in SSC conditions with RA was predominantly increased up to day 3 and decreased by day 5. Meanwhile, we tested the expression of another two pluripotent genes, *Oct4* and *Nanog*, which have been reported to express in proliferating germ cells but not mature spermatogonia [36]. Our results showed that *Oct4* and *Nanog* down-regulated during differentiation (Figure 3I,J), indicating that cells were at differentiation stage of spermatogonia. Overall, our data suggest that cells underwent meiosis during mouse ESCs differentiation in SSC conditions with RA.

The article "Retinoic acid combined with spermatogonial stem cell conditions facilitate the generation of mouse germ-like cells" was published in 2017. Journal: Biosci Rep.

### RA combined with SSC conditions yield Acrosin-positive cells

To further examine whether post-meiotic cells are generated during mouse ESCs differentiation in SSC conditions with RA. We first measured the mRNA level of polar Acrosin, which is a specific marker for post-meiotic cells [37]. As expected, we observed a dramatic increase in *acrosin* expression in SSC conditions with RA compared with ESC medium or SSC conditions without RA (Figure 4A) and exhibited polar Acrosin localization (Figure 4B) at day 6, suggesting a number of post-meiotic cells appearing during differentiation.

**Figure 4:** RA enables the generation of Acrosin-positive cells (**A**) QPCR results of *acrosin* expression at day 0, 3, 5 and 6 during mouse ESCs differentiation. The expression levels of mRNA were normalized to *β-actin*, and expressed as a ratio of mRNA levels of genes of interest to that of *β-actin*. Values with * show significant differences among various treatments at the indicated time points (***, *P*<0.001). (**B**) Immunofluorescence staining with Acrosin at day 0, 3 and 6 during mouse ESCs differentiation in SSC conditions with RA. Scale bar, 100 μm. (**C**) FACS analysis of Acrosin-positive cells in SSC conditions with or without RA.

To further confirm this result, we analysed differentiated cells at day 6 in SSC conditions with or without RA by FACS. Our result showed that Acrosin-positive cells were approximately 17.2% (Figure 4C). Overall, our data suggest that a small subpopulation of Acrosin-positive, post-meiotic cells appear during differentiation in SSC conditions with RA.

## Discussion

Recently, many studies reported that germ cells could be stably achieved *in vitro* through inducing PSCs with a set of combination of BMP4/4b, SCF, LIF and EGF [7] or SSC conditions [13]; furthermore, Zhou et al. [9] reported that co-culture of PGC-like cells with neonatal testicular somatic cells and sequential exposure to several hormones yielded haploid cells and further fertile offspring. However, direct and efficient induction system of spermatogenic cells is still partially incomplete. In the present study, our results indicated that RA combined with SSC conditions contained a set of soluble factors such as bFGF and GDNF could directly induce mouse ESCs into germ-like cells and with the effect of RA could promote the differentiation efficiency, whereas SSC conditions solely was insufficient in mouse spermatogenic conversion process (Figure 2).

The article "Retinoic acid combined with spermatogonial stem cell conditions facilitate the generation of mouse germ-like cells" was published in 2017. Journal: Biosci Rep.

It is worth noting that human and mouse PSCs are indeed representing two different metastable pluripotent states, termed as ‘primed’ and ‘naïve’ states [21] and naïve state has higher pluripotency potential compared with primed state. Recently, Surani and Hanna group showed highly efficient differentiation of human naïve PSCs into primordial stem cells [38]; however, spermatogenic cells have not yet derived from human naïve PSCs so far. In this regard, our work on mouse ESCs is important since it may provide insights that can be potentially useful for the generation of human germ cells directly from naïve PSCs.

Previous researches have reported that PGCs, the germ cell progenitor, undergo migration, proliferation and differentiation into spermatogenic lineage during development *in vivo* [5]. Our results showed that the expression of two PGCs markers, *Prdm14* and *Stella* were notably increased from day 5 to day 6 (Figure 3A,B) in SSC conditions with RA; in addition, it has been reported that during embryogenesis, the pluripotency gene *Sox2* represses the expression of germ-line genes in inner cell mass [32], and is slightly down-regulated in epiblast, which contributes to competency for PGCs, but thereafter *Sox2* is significantly regained in PGCs and supports proliferation of PGCs [7,33]; our results showed that the expression of *Sox2* in SSC conditions with RA was slightly decreased at day 3 and increased from day 3 to 6 (Figure 3C), which is consistent with previous reports [7,33]; overall, our results indicated that cells undergo a differentiation progress of PGCs stage.

It has been reported that RA dramatically stimulates *Stra8* expression in undifferentiated spermatogonia but has a less impact on differentiating spermatogonia [17]. In the present study, our QPCR results (Figure 3G) showed that the expression of *Stra8* in SSC conditions with RA was predominantly increased up to day 3 and decreased by day 5, meanwhile, the expression of *acrosin* that first appeared in the haploid cells and was synthesized only in the post-meiotic stages of spermatogenesis [39], was markedly up-regulated from day 3 to day 6 in SSC conditions with RA (Figure 4A), which is consistent with previous observations by West et al. [40] and Geijsen et al. [22]. In addition, *Scp1*, involved in the meiotic prophase in chromosome rearrangements [34]; similarly, highly expressed over first 5 days. These results suggest that the collective effects of RA and SSC conditions promote the expression of *Stra8*, *acrosin* and *Scp1* to facilitate the initiation of differentiation. Besides, MVH protein, a marker for PGCs and specific for differentiating germ cells from the late migration stage to the post-meiotic stage [41], was detected during differentiation (Figure 2B), which is consistent with the observation by Hayashi et al. [7]. Moreover, Acrosin was detected at day 3 and highly expressed at day 6 (Figure 4B), which was similar to the immunostaining results of MVH and DAZL (Figure 2B,C), suggesting that ESCs start to form post-meiotic cells at day 3 by SSC conditions with RA treatment and are undergone meiosis during mouse ESCs differentiation.

The article "Retinoic acid combined with spermatogonial stem cell conditions facilitate the generation of mouse germ-like cells" was published in 2017. Journal: Biosci Rep.

In the present study, our data showed that RA promoted spermatogenesis of mouse naïve PSCs. The role of RA in the regulation of naïve pluripotency and spermatogenesis seems to be interesting for further study. Indeed, researchers have realized RA is an important player in stem cell identity. For example, RA has been used to iPSCs differentiation towards neural ectoderm lineage [42]. In addition, RA could promote mouse ESCs differentiating into PGCs and SSCs [22,24]. One possible role of RA during differentiation may be to preserve cell viability. For example, previous studies have shown that RA is a mitogen which can stimulate PGC survival *in vitro* [43] and prevent PGCs from apoptosis *in vivo* [43]. Moreover, RA can stimulate PGCs proliferation *in vitro* in serum with LIF of mouse ESC conditions [43]. Further study should investigate the interplay between extracellular signals, cell survival and cell identity control.

In summary, our work provides a good approach for germ-like cell differentiation from mouse ESCs and suggests RA to be a promising additive for improving the differentiation potential of other types of stem cells. RA has been shown to activate many endogenous genes in a cell type-specific manner [16–18], therefore, it is tempting to speculate that addition of RA may also improve various types of cell fate conversions [44].

## Abbreviations

AP: alkaline phosphatase
BMP: bone morphogenetic protein
ESCs: embryonic stem cells
GDNF: glial cell line-derived neurotrophic factor
hiPSCs: human induced pluripotent stem cells
iPSCs: induced pluripotent stem cells
PGCs: primordial germ cells
PSCs: pluripotent stem cells
QPCR: quantitative real-time PCR
RA: retinoic acid
RT: room temperature
SSC: spermatogonial stem cell
KSR: knockout serum replacement
NEAA: non-essential amino acids
bFGF: basic fibroblast growth factor
LIF: leukemia inhibitory factor
PE: phycoerythrin
